# Vitamin D and iodine status was associated with the risk and complication of type 2 diabetes mellitus in China

**DOI:** 10.1515/biol-2021-0019

**Published:** 2021-02-18

**Authors:** Yafen Zhuo, Lin Ling, Zhichun Sun, Wensen Huang, Zhenzhen Hong, Yaping Zhang, Xuefeng Peng, Xiaoyu Liu, Weilan Yuan, Wang-Yang Xu, Yi Zhang

**Affiliations:** Department of Endocrinology, Quanzhou First Hospital Affiliated to Fujian Medical University, No. 250, East Street, Licheng District, Quanzhou, 362300, Fujian, China; Department of Internal Medicine, Quanzhou Medical College, Quanzhou, 362300, China; Department of Oncology, Quanzhou First Hospital Affiliated to Fuji Medical University, Quanzhou, 362300, China; Department of Information Technology, Biotecan Medical Diagnostics Co., Ltd, Zhangjiang Center for Translational Medicine, Shanghai, 201204, China; Medical Department, Singlera Genomics Inc., Lane 500, Furonghua Road, Pudong New District, Shanghai, 201318, China

**Keywords:** 25(OH)D level, vitamin D, urinary iodine concentration, type 2 diabetes mellitus, T2DM risk, a prediction model

## Abstract

The purpose of this study was to assess the relationship between 25-hydroxyvitamin D (25(OH)D), urinary iodine concentration (UIC), and type 2 diabetes mellitus (T2DM) risk and complications and to establish a model to predict T2DM in the general population. A total of 567 adults (389 T2DM patients and 178 controls) were enrolled, and the levels of 25(OH)D, iodine, and blood biochemical parameters were measured. Pearson’s correlation analysis showed an inverse correlation between 25(OH)D level, UIC, and T2DM risk. Low 25(OH)D level was a risk factor for developing T2DM (OR, 0.81; 95% CI, 1.90–2.63; *P* = 0.043) after adjustment for multiple risk factors. 25(OH)D level and UIC were inversely correlated with short-term and long-term glucose levels. 25(OH)D deficiency was also associated with a high incidence of T2DM complicated with thyroid dysfunction. A prediction model based on 25(OH)D, iodine status, and other risk factors was established and recommended to screen high-risk T2DM in the general population and provide early screening and timely treatment for them.

## 1 Introduction

Diabetes mellitus is a widespread metabolic disorder. In China, approximately 11% of the population has diabetes according to the latest reports [1,2]. The pathogenesis of type 2 diabetes mellitus (T2DM) includes relatively insufficient insulin secretion and insulin resistance [3,4]. The effects of nutritional risk factors on islet β-cell physiology, especially insulin secretion, have attracted great attention [5]. Avoiding β-cell dysfunction by regulating nutrients becomes an effective way to prevent diabetes. The immune system is an important defense mechanism to maintain health. The effect of diet on various aspects of the immune system has always been studied. It has been reported that different types of proteins in diet directly affect the innate response of B lymphocytes to immunogenic stimulation [6]. In particular, high fat or high carbohydrate daily diet would decrease B lymphocytes, while the number of pancreatic CD20 + B cells was related to the loss of β cells, indicating an important role of diet regulation of B cells and islet β cells in the occurrence and development of diabetes mellitus [7,8].

Vitamin D, a secosteroid hormone, contributes to calcium homeostasis and works primarily in the musculoskeletal system [9]. In addition, vitamin D plays a major role in physiological processes associated with multiple chronic diseases such as diabetes mellitus [10,11]. Recent evidence from human and animal research have shown the relationship between vitamin D status and glucose homeostasis as well as impaired insulin sensitivity [12,13,14,15,16]. Many epidemiological studies showed that vitamin D deficiency was common in diabetes subjects [17,18,19], while some trials indicated that 25-hydroxyvitamin D (25(OH)D) levels had no influence on the incidence of diabetes [20,21].

Iodine is a major component of the thyroid hormone [22]. For T2DM, thyroid hormones are determinants of glucose homeostasis [23,24]. It is reported that thyroid disease occurs more frequently in diabetic patients than in the general population [25]. Both thyroid disorders and DM would mutually affect and interconnect with each other [26,27]. Thyroid hormones could influence glucose metabolism and hyperthyroidism, which has been proved to act as an important factor contributing to hyperglycemia [28]. About one-third of the population is at risk of iodine deficiency-related diseases because of iodine-deficient diet and environment. The adoption of universal salt iodization (USI) has been widespread since the 1990s in the world. Located in China, Quanzhou is a southern coastal city with abundant sunshine almost throughout the year, and the local diet is rich in iodine because people mainly consume seafood and milk. However, little is known about whether vitamin D and iodine status plays an important role in the incidence and process of T2DM.

In the present study, we sought to assess the relationship between vitamin D and iodine status and T2DM in Chinese population living in Quanzhou and then provided a prediction model to screen high risk of T2DM among individuals.

## 2 Materials and methods

### 2.1 Study population

From November 2017 to February 2019, a total of 389 newly diagnosed T2DM patients were enrolled from First Hospital of Quanzhou City, Fujian Province, China. The diagnosis of T2DM followed the World Health Organization definition. Participants were selected based on the following criteria: negative to (1) history of neoplasm, (2) history of any mental disorder, (3) history of diabetes, (4) history of thyroid cancer or thyroidectomy, (5) history of drug abuse, and (6) history of taking the drug to treat diabetes or thyroid diseases. The number of subjects (178) who passed a medical evaluation including a complete physical examination to exclude the existence of T2DM and thyroid diseases was considered as the control group. All samples were collected in summer and autumn. Clinical information including age, gender, body mass index (BMI), familiar history of T2DM or thyroid diseases, dietary habits, and taking iodized salt in diet were filled in. Influence of diet, including seafood (three groups: no seafood consumption; occasional: one to two meal containing seafood per week on average; frequent: at least three meal containing seafood per week) and cow’s milk (three groups: no consumption; occasional: 1–500 mL per week on average; frequent: at least 500 mL per week), was recorded according to the above classification.


**Informed consent:** Informed consent has been obtained from all individuals included in this study.
**Ethical approval:** The research related to human use has been complied with all the relevant national regulations and institutional policies, and in accordance with the tenets of the Helsinki Declaration and has been approved by the Ethics Committee of Fujian Medical University.

### 2.2 Laboratory examinations

Fasting blood sample (8 h overnight) was drawn into a serum separator tube which was centrifuged (3,000 rpm, 15 min, 4°C) to separate serum (used for measuring fasting glucose, fructosamine, C peptide, lipid profiles, serum creatinine, thyroid hormones, and thyroid antibodies). Detection values of serum glucose, glycosylated hemoglobin (HbA1c), fructosamine, C peptide, lipid profiles, serum creatinine, thyroid hormones including serum-free thyroxine (FT4), free triiodothyronine (FT3), and thyroid-stimulating hormone (TSH) were determined using an automatic biochemical analyzer (Beckman Coulter, Inc., CA, USA). The measurement of antibodies, including thyroid peroxidase antibodies (TPOAb), thyroglobulin antibodies (TGAb) and thyroid-stimulating hormone receptor antibodies (TRAb), and thyroglobulin was determined using an automatic biochemical analyzer (Roche Ltd, Switzerland). Thyroid antibodies were deemed as positive when they were above the normal range. C-reactive protein (CRP) was detected using an automatic detector (Lifotronic, China). HbA1c was measured by a glycosylated hemoglobin analyzer (Arkray Inc., Japan). Reference ranges are reported in Table A1. The diagnosis of thyroid dysfunction was made according to the following definitions:

1. Clinical hyperthyroidism (any one of the below criteria): decreased TSH with elevated FT4 and/or elevated FT3; patients with a history of hyperthyroidism who were receiving anti-thyroid agents.
2. Clinical hypothyroidism: elevated TSH with decreased FT4; patients with a history of hypothyroidism who were receiving levothyroxine.
3. Subclinical hyperthyroidism: decreased TSH with normal FT4
4. Subclinical hypothyroidism: elevated TSH with normal FT4

### 2.3 Serum 25(OH)D level and UIC measurement

The serum 25(OH)D levels were measured by an automatic biochemical analyzer (Roche Ltd, Switzerland). According to the National standard, a serum 25(OH)D level of <10 ng/mL was defined as a severe deficiency; <20 ng/mL as a deficiency; from 20 to 30 ng/mL insufficiency; and >30 ng/mL as 25(OH)D sufficiency. The urine specimen was collected from all participants. UIC was detected by inductively coupled plasma mass spectrometry (Agilent Technologies, Inc., Tokyo, Japan) as described in a previous study [29]. According to the National standard, UIC < 100 μg/L was defined as a deficiency, from 100 to 300 μg/L adequate, and >300 μg/L as excess.

### 2.4 Logistic regression model

Several typical and recent artificial intelligence algorithms were established in the context of T2DM, and the logistic regression model became our base model. Logistic scores to predict T2DM risk probability in the Chinese population were obtained according to the following equation:

\text{T}2\text{DM}\hspace{.5em}\text{risk}\hspace{.5em}\text{probability}=\frac{{\text{e}}^{\left({\beta }_{0}+\sum {\beta }_{i}{X}_{i}\right)}}{1+{\text{e}}^{\left({\beta }_{0}+\sum {\beta }_{i}{X}_{i}\right)}},

where *β*_0_ is the constant, while *β*_*i*_ is the coefficient of variable *X*_*i*_. *X*_*i*_ = 1 means a categorical risk factor is present and 0 means a categorical risk factor is absent. Data are shown as area under the curve (AUC) and receiver operating characteristic curve.

### 2.5 Statistical analysis

Statistical analysis was done using Python software (Version 3.6). Categorical variables were shown as numbers with percentages (%). Continuous variables were presented as mean ± standard deviation. Correlation analyses were performed using the Pearson’s correlation method. Multivariate logistic regression analysis was conducted to assess the risk factors for T2DM. Kruskal–Wallis *H* test was used to analyze intra-group or inter-group differences. The level of significance was set at *P* < 0.05.

## 3 Results

### 3.1 General characteristics of participants

Age, fasting glucose, fructosamine, HbA1c, total cholesterol (TC), triglyceride (TG), low-density lipoprotein cholesterol (LDL-C), TSH, and thyroglobulin were markedly increased in T2DM patients compared to the controls (*P* < 0.001). The levels of 25(OH)D, iodine, high-density lipoprotein cholesterol (HDL-C), creatinine, FT4, and FT3 were significantly decreased in the T2DM group than those in the controls (*P* < 0.05). The positive rates of TPOAb, TRAb, and TGAb were significantly higher in the diabetic patients than those in the control group (*P* < 0.05). According to the questionnaire responses, the number of T2DM patients who ate seafood frequently was lower than that of the control group, and the number of people who never ate seafood was higher than that of the controls. The numbers of T2DM patients who consumed milk frequently and who never drink milk were both higher than the controls. Of the T2DM patients, 43.70 and 41.57% of the controls consumed iodized salt (Table 1).

**Table 1:** General characteristics of T2DM and the controls

	T2DM (*n* = 389)	Control (*n* = 178)	*P*-value
Age (years)*	51.83 ± 12.70	47.03 ± 11.47	<0.001
Gender (male/female)	245/144 (62.98/37.02)	103/75 (57.87/42.13)	0.196
BMI (kg/m^2^)*	24.23 ± 4.38	23.86 ± 2.99	0.241
25(OH)D (ng/mL)*	20.53 ± 5.46	24.85 ± 5.97	<0.001
UIC (μg/L)*	158.6 ± 92.46	212.15 ± 86.65	<0.001
Glucose (mmol/L)*	10.87 ± 3.69	5.54 ± 0.87	<0.001
Fructoseamine (mmol/L)*	3.27 ± 0.74	2.21 ± 0.34	<0.001
HbA1c (%)*	9.61 ± 2.61	5.3 ± 0.66	<0.001
C peptide (μg/L)*	2.19 ± 1.13	2.19 ± 0.7	0.977
TC (mmol/L)*	5.31 ± 1.33	4.73 ± 0.9	<0.001
TG (mmol/L)*	2.06 ± 1.44	1.47 ± 0.6	<0.001
LDL-C (mmol/L)*	3.38 ± 1.08	3.03 ± 0.71	<0.001
HDL-C (mmol/L)*	1.12 ± 0.28	1.32 ± 0.24	<0.001
Creatinine (μmol/L)*	75.89 ± 30.95	85.99 ± 18.82	<0.001
CRP (mg/L)*	3.59 ± 1.57	3.29 ± 2.68	0.106
FT4 (ng/mL)*	0.98 ± 0.47	1.22 ± 0.69	<0.001
FT3 (μg/dL)*	5.04 ± 1.00	5.22 ± 0.98	0.039
TSH (uIU/mL)*	2.22 ± 1.74	1.29 ± 0.85	<0.001
TPO-antibody positivity	36 (11.69)	6 (4.48)	0.028
TR-antibody positivity	40 (12.99)	1 (0.75)	<0.001
TG-antibody positivity	19 (6.17)	0 (0.0)	0.007
Thyroglobulin (μg/L)*	15.39 ± 18.57	9.49 ± 5.92	<0.001
Sea food (fish, crab, and shrimp)			
Frequent	68 (17.48)	48 (26.96)	0.006
Occasional	288 (74.04)	130 (73.04)	
Never	33 (8.48)	0 (0.00)	
Cow’s milk			
Frequent	23 (5.91)	1 (0.56)	<0.001
Occasional	148 (38.05)	148 (83.15)	
Never	218 (56.04)	29 (16.29)	
Iodized salt			
Yes	170 (43.70)	74 (41.57)	0.635
No	219 (56.30)	104 (58.43)	
Sampling season			
Summer	205 (52.70)	79 (44.38)	0.066
Fall	184 (47.30)	99 (55.62)	

Categorical variables are presented as numbers and percentage (%). Continuous variables presented as mean ± standard deviation (SD) are marked with asterisk (*).

### 3.2 Correlation between clinical variables and T2DM risk

Pearson’s correlation analysis was conducted to find the correlation of clinical risk factors and the presence of T2DM (Figure 1). There is a positive and significant correlation between T2DM risk and the levels of HbA1c (*r* = 0.67, *P* < 0.001), fasting glucose (*r* = 0.62, *P* < 0.001), fructosamine (*r* = 0.61, *P* < 0.001), age (*r* = 0.36, *P* < 0.001), TC (*r* = 0.22, *P* < 0.001), gender (*r* = 0.19, *P* < 0.001), LDL-C (*r* = 0.16, *P* < 0.001), and TG (*r* = 0.13, *P* = 0.04). Significant inverse correlations between T2DM risk and 25(OH)D (*r* = −0.34, *P* < 0.001), HDL-C (*r* = −0.33, *P* < 0.001), UIC (*r* = −0.26, *P* < 0.001), and creatinine (*r* = −0.17, *P* < 0.001) were found in the study.

**Figure 1:** Pearson’s correlation between clinical factors and T2DM risk.

### 3.3 Low 25(OH)D level was a risk factor for developing T2DM

The etiology of T2DM is complex. Clinical factors such as HbA1c, fructosamine, and dyslipidemia are considered traditional risk factors for T2DM. In this study, T2DM was used as a variable response and risk factors as explanatory variables in the multivariate logistic regression. We found that low 25(OH)D level was deemed as a risk factor after additional adjustment for other risk factors. Elevated fasting glucose and HbA1c were risk factors for T2DM (Table 2).

**Table 2:** Multivariable logistic regression analysis of risk factors for T2DM

Variables	*β*	SE	Wald *χ* ^2^	OR value	95.0% CI for *β*	*P*-value
Age	0.06	0.04	1.53	1.06	0.99–1.16	0.127
25(OH)D	−0.21	0.10	−2.02	0.81	0.64–0.97	0.043
UIC	0.01	0.01	2.62	1.01	1.00–1.03	0.009
Glucose	1.80	0.48	3.77	6.05	2.85–19.70	<0.001
Fructoseamine	2.00	1.14	1.76	7.38	0.96–98.81	0.079
HbA1c	2.98	0.86	3.45	19.60	5.27–171.45	<0.001
TC	0.78	0.50	1.53	2.15	0.82–6.55	0.126
TG	1.10	0.82	1.34	3.01	0.62–15.77	0.181
Creatinine	−0.04	0.02	−2.39	0.96	0.90–0.99	0.017

OR, odds ratio; CI, confidence interval.

### 3.4 Effects of 25(OH)D level and UIC on short-term and long-term glucose level

Inverse correlations between 25(OH)D level, UIC and fasting glucose, fructosamine and even HbA1c were observed (*P* < 0.0001). 25(OH)D level was negatively associated with TC, TG, and LDL-C, while positively associated with HDL-C (Table A2).

### 3.5 25(OH)D deficiency contributed to the incidence of TD in T2DM

As shown in Table 3, serum 25(OH)D deficiency was not only associated with the incidence of T2DM (no TD) (45.26 vs 24.16%, *P* = 0.002) but also significantly associated with the incidence of TD in T2DM (62.90 vs 45.26%, *P* = 0.012). Hypothyroidism and subclinical hypothyroidism were more common in the 25(OH)D-deficient group (Table A3). In accordance with these, a significant inverse correlation between 25(OH)D level and TSH in T2DM group was observed (Table A2). Iodine deficiency was significantly associated with the incidence of T2DM (35.17 vs 9.27%, *P* < 0.001), but it had no correlation with the prevalence of TD in T2DM (27.42 vs 35.17%, *P* = 0.843). Iodine excess was not associated with the risk of T2DM (8.56 vs 15.95%, *P* = 0.628), but it contributed to the incidence of TD (25.81 vs 8.56%, *P* = 0.003). Hypothyroidism was the most common disorder of thyroid dysfunctions in the UIC excess group, whereas subclinical hypothyroidism was most common in the UIC-deficient group (Table A4). UIC was found to have a significant positive correlation with TSH (Table A2).

**Table 3:** Incidence of TD according to 25(OH)D and iodine levels

	T2DM with TD	T2DM without TD	Controls	*P*-value	*P*-value
	(1)	(2)	(3)	(1) vs (2)	(2) vs (3)
25(OH)D level					
Deficiency	39 (62.90)	148 (45.26)	43 (24.16)	0.012	0.002
Non-deficiency	23 (37.10)	179 (54.74)	135 (75.84)		
UIC					
Deficiency	17 (27.42)	115 (35.17)	14 (9.27)	0.843	<0.001
Adequate	29 (46.77)	184 (56.27)	137 (90.73)		
UIC					
Excess	16 (25.81)	28 (8.56)	26 (15.95)	0.003	0.628
Adequate	29 (46.77)	184 (56.27)	137 (84.05)		

Categorical variables are presented as numbers and percentage (%).

Chi-square test was used to calculate the difference between groups.

### 3.6 A model for predicting the T2DM risk

A logistic regression model based on multiple clinical variables for assessing the risk of T2DM was built. Conventional risk factors, such as HbA1c, glucose, fructosamine, UIC, creatinine, TC, BMI, 25(OH)D level, age, TG, LDL-C, and C peptide, were incorporated into the model (ranking by the feature importance of variables in the model). As shown in Figure 2, the AUC was 0.95 for the test set. It was superior to the model without 25(OH)D level (AUC = 0.92) (Figure A1a) and the model without UIC (AUC = 0.86) (Figure A1b). When both 25(OH)D and UIC were not included, the AUC of the model was 0.83 (Figure A1c). Model score output was positively correlated with the risk of T2DM in the general population.

**Figure 2:** A prediction model for screening the high-risk T2DM in the population.

## 4 Discussion

In this study, we found that vitamin D and iodine levels were much lower in T2DM patients than that in control subjects. The prevalence of vitamin D deficiency in T2DM patients was 48% but the control was 24%. This study also showed an iodine deficiency in 34% of the T2DM cases and about 8% in the controls. Quanzhou is a southern coastal city with abundant sunshine almost throughout the year, and the diet rich in vitamin D and iodine, due to local people’s preference of seafood and milk. Besides moreover, China has greatly improved iodine consumption levels resulting from the government implementation of the USI policy in 1996 [30]. However, this finding showed that vitamin D and iodine levels were still deficient in coastal cities of China, despite inherent environmental advantages.

This study reported a reduction in 25(OH)D and iodine level in a Chinese population before the onset of T2DM. Significant inverse correlations between 25(OH)D, UIC, and T2DM risk were found. Multivariate logistic regression models further revealed that low 25(OH)D level was a risk factor for the onset of T2DM in the Chinese population, suggesting that 25(OH)D contributed to the pathophysiology of T2DM. Similar to our results, several observational studies have shown that 25(OH)D status was significantly lower in T2DM or people with impaired glucose tolerance [31,32,33,34]. The effect of decreased vitamin D levels on increasing T2DM risks was because of an increase in insulin resistance [35,36]. 1,25-Dihydroxyvitamin D can induce pancreatic β cell to secrete insulin and also elevate the expression of the insulin receptors, so as to increase the response to glucose [37,38]. Therefore, early correction of vitamin D levels in the high-risk population has a positive effect on the prevention of T2DM.

Besides, low 25(OH)D level was related to a high risk of diabetic complications including peripheral neuropathy, nephropathy, and thyroid diseases. The prevalence of TD was significantly higher in the serum 25(OH)D-deficiency group (20.86%) than that in the 25(OH)D insufficiency and sufficiency groups (11.48 and 10.53%, respectively). Therefore, the prevention of vitamin D deficiency is of great significance for preventing diabetes and for clinical monitoring of thyroid gland function. Further studies are required to focus on the effects of vitamin D levels on the pathogenesis of thyroid dysfunction and whether the occurrence and progression of thyroid diseases would be modulated by vitamin D supplementation in subjects with excessive iodine intake.

Another nutrient, iodine, was negatively correlated with T2DM risk. Although iodine plays great roles in multiple diseases, the role of iodine in T2DM risk was less studied. In this study, we showed that UIC was decreased in T2DM when compared to the controls. A recent study conducted in a Chinese population demonstrated that TSH had a positive correlation with the iodine/creatinine ratio, and a positive correlation between TSH and insulin resistance was observed. It is known that thyroid hormones regulate lipid metabolism and cause increased weight gain and insulin resistance, but this speculation has also been questioned due to the reports of alterations in thyroid hormones having the possible consequence of increased weight gain [39]. In this study, although UIC was negatively correlated with T2DM risk through Pearson’s correlation analysis, we found that low UIC was not a risk factor for T2DM in multivariate logistic regression analysis. In addition, iodine deficiency was associated with an increased incidence of T2DM but not with TD. Iodine excess was only associated with a high prevalence of TD in T2DM patients but not with the incidence of T2DM.

Considering the joint evaluated values of clinical parameters in predicting T2DM, a clinical model was constructed to predict the risk of T2DM. 25(OH)D, UIC, glucose, HbA1c, and other variables were input in the model as variables, and the corresponding probability of risk can be output. An AUC = 0.95 of the model exhibited its advantage, and this digital model can help clinicians to provide prevention and early intervention measures for T2DM patients. Because T2DM is associated with a combination of multiple risk factors, we believe that multiple risk factors together could predict the risk more effectively than single risk factors such as glucose or HbA1c. Compared with the model without 25(OH)D and/or UIC, this model was superior, which indicated that the serum 25(OH)D level and UIC had great significance for the detection of T2DM. We thereby suggest that nutrition modulation, including vitamin D, iodine, and other elements related to glucose homeostasis and insulin sensitivity, plays a vital and objective role in the occurrence and development of prediabetes or T2DM in Chinese individuals.

Significant inverse correlations between 25(OH)D, UIC, and short- and long-term glucose levels suggested a critical role of 25(OH)D and iodine in the development of impaired glucose homeostasis. HbA1c which represents the blood glucose status of 2–3 months is the “gold standard” for evaluating long-term blood glucose control. Thus, the early detection and correction of vitamin D levels in high-risk people may play a beneficial role in the occurrence and development of prediabetic blood glucose abnormalities. There are some limitations in this study. First, insulin sensitivity, resistance, and β-cell function were not detected in this study. Second, although all blood samples were collected in summer and autumn, there was no significant difference in 25(OH)D level between summer and autumn. There was no in-depth analysis of the impact of seasons on the results. Third, the effect of sunshine duration and sunscreen use on 25(OH)D level was not analyzed. Fourth, this is a single-center study involving almost the same Han population in the same region and the sample size was relatively small.

## 5 Conclusion

This study illustrated inverse associations between 25(OH)D level, UIC, and the risk of T2DM. In addition, low 25(OH)D level was a risk factor for T2DM and 25(OH)D deficiency was associated with the incidence of TD in T2DM. A prediction model was constructed to help clinicians better prevent T2DM. Thus, monitoring 25(OH)D and iodine levels is of great significance for maintaining glucose metabolism and preventing T2DM progression.

## Figures and Tables

**Figure A1:** Established models for the prediction of T2DM risk. (a) The prediction model without 25(OH)D level. (b) The prediction model without UIC. (c) The prediction model without 25(OH)D level and UIC.

## Appendix

**Table A1:** Biochemical indicators and reference range

Indexes	Reference range
Glucose (mmol/L)	3.89–6.11
Fructoseamine (mmol/L)	1.7–2.5
HbA1c (%)	4–6
C peptide (μg/L)	1.1–4.4
TC (mmol/L)	3.6–5.17
TG (mmol/L)	0.4–2.3
LDL-C (mmol/L)	1.5–3.4
HDL-C (mmol/L)	1.04–1.55
CRP (mg/L)	≤8
Creatinine (μmol/L)	44–133
Free T4 (ng/mL)	0.87–1.78
Free T3 (μg/dL)	4.5–12.23
TSH (uIU/mL)	0.34–5.6
TPO-antibody (KIU/L)	0–34
TR-antibody (IU/L)	0–1.75
TG-antibody (KIU/L)	0–115
Thyroglobulin (μg/L)	3.5–77

**Table A2:** Correlation between urinary iodine concentration and serum 25(OH)D level

	*r*	*P*-value
T2DM	−0.03	0.617
Control	0.12	0.109

**Table A3:** Correlation between 25(OH)D level, UIC, and clinical factors

	25(OH)D level		UIC	
	*r*	*P*-value	*r*	*P*-value
Age (years)	−0.04	0.241	−0.03	0.406
Gender (male/female)	0.01	0.737	−0.07	0.096
BMI (kg/m^2^)	−0.02	0.662	0.00	0.913
Glucose (mmol/L)	−0.32	<0.0001	−0.59	<0.0001
Fructoseamine (mmol/L)	−0.21	<0.0001	−0.20	<0.0001
HbA1c (%)	−0.23	<0.0001	−0.21	<0.0001
C peptide (μg/L)	−0.02	0.650	0.00	0.908
TC (mmol/L)	−0.11	0.012	−0.07	0.090
TG (mmol/L)	−0.14	0.001	−0.09	0.032
LDL-C (mmol/L)	−0.10	0.020	−0.05	0.210
HDL-C (mmol/L)	0.11	0.007	0.05	0.215
Creatinine (μmol/L)	−0.05	0.200	0.07	0.112
Free T4 (ng/mL)	0.07	0.095	0.07	0.078
Free T3 (μg/dL)	0.08	0.121	−0.02	0.724
TSH (uIU/mL)	−0.14	0.006	0.18	0.000

**Table A4:** Prevalence of TD according to 25(OH)D level in T2DM

	25(OH)D level		
	Deficiency (*n* = 187)	Insufficiency (*n* = 183)	Sufficiency (*n* = 19)
Total			
Euthyroid	148 (79.14)	162 (88.52)	17 (89.47)
Thyroid dysfunction	39 (20.86)	21 (11.48)	2 (10.53)
Subtypes			
Hyperthyroidism	1 (0.53)	3 (1.64)	0
Hypothyroidism	22 (11.76)	5 (2.73)	1 (5.26)
Subclinical hyperthyroidism	1 (0.53)	2 (1.09)	0
Subclinical hypothyroidism	15 (8.02)	11 (6.01)	1 (5.26)

TD, thyroid dysfunction.

Categorical variables are presented as numbers and percentage (%).

**Table A5:** Prevalence of TD according to UIC in T2DM

	UIC		
	Deficiency (*n* = 132)	Adequate (*n* = 213)	Excess (*n* = 44)
Total			
Euthyroid	115 (87.12)	184 (86.38)	28 (63.64)
Thyroid dysfunction	17 (12.88)	29 (13.62)	16 (36.36)
Subtypes			
Hyperthyroidism	1 (0.76)	2 (0.94)	2 (4.55)
Hypothyroidism	3 (2.27)	13 (6.10)	12 (27.27)
Subclinical hyperthyroidism	2 (1.52)	1 (0.47)	0
Subclinical hypothyroidism	11 (8.33)	13 (6.10)	2 (4.55)

TD, thyroid dysfunction.

Categorical variables are presented as numbers and percentage (%).
